# Comparison of complications in one-stage bilateral total knee arthroplasty with and without drainage

**DOI:** 10.1186/s13018-014-0140-1

**Published:** 2015-01-14

**Authors:** Ning Li, Ming Liu, Dan Wang, Mang He, Lei Xia

**Affiliations:** Department of Orthopedics, The First Affiliated Hospital of Zhengzhou University, 1 Jianshe Road, Zhengzhou, 450052 China

**Keywords:** Drainage, One-stage, Bilateral, Total knee arthroplasty, Randomized controlled trials

## Abstract

**Purpose:**

The aim of this meta-analysis was to compare the complication rates of one-stage bilateral total knee arthroplasty (TKA) with and without drainage in order to identify whether there was no clinical significance and the value of drainage.

**Methods:**

Randomized controlled trials (RCTs) based on bilateral TKA with and without drainage were identified via a search of PubMed, EMBASE, Cochrane Central Register of Controlled Trials, Wanfang databases, and Google Scholar, which were published up to May 2014. Methodological quality was assessed by the Physiotherapy Evidence Database scale. After data extraction, we compared the outcomes using fixed-effects or random-effects models depending on the heterogeneity.

**Results:**

Three RCTs involving 125 one-stage bilateral TKA patients with an average follow-up of 14 months met the predetermined inclusion criteria. There were 56 total complications in TKA without drainage and 17 with drainage. Except for less erythema and ecchymosis around the wound in the drainage group, there were no statistical differences in wound healing, wound infection, swelling, and deep vein thrombosis in one-stage bilateral TKA with and without drainage.

**Conclusion:**

The current evidences confirm that both drainage and non-drainage have similar clinical value in one-stage bilateral TKA. However, the conclusion should be used with caution due to the limitations of the current study.

## Introduction

Total knee arthroplasty (TKA) is a standardized highly successful procedure in treating late osteoarthritis (OA) and rheumatoid arthritis (RA) of knee joints. Drainage is frequently used with the purpose of preventing hematoma accumulation, decreasing the risk of infection, and delaying wound healing in TKA [1]. However, some studies claimed that there was no difference in healing of wounds, postoperative blood transfusions, complications, or range of motion in primary TKA [2-4]. What needs to be noted is that the above findings were based on unilateral TKA, and there may be possible influences of age, sex, systemic disease, reaction to anticoagulants or other medications, and effort and differences in rehabilitation.

Until now, no meta-analyses based on bilateral TKA were conducted to evaluate the clinical efficacy and safety of drainage. Therefore, it is necessary to have a latest, up-to-date meta-analysis to investigate this issue. In the current study, we performed a systematic review and meta-analysis of randomized controlled trials (RCTs) to compare complication rates of one-stage bilateral TKA with and without drainage in order to identify the clinical significance and value of drainage.

## Methods

### Literature search

Electronic databases (MEDLINE, EMBASE, Cochrane Central Register of Controlled Trials, Wanfang Data, and Google Scholar) were searched for RCTs which were published up to May 2014 without limits by two independent reviewers. The search terms were “drainage” or “drain,” “total knee arthroplasty” or “total knee replacement,” and “bilateral” and “randomized controlled trial”. We also searched the reference lists of related reviews and original articles identified for any relevant trials including clinical trials and RCTs involving adult humans.

### Eligibility criteria

Studies were identified according to the following criteria: (1) the study was based on one-stage bilateral TKA, (2) a suction drainage was placed by randomization in only one knee for all patients, with the other knee as self-control, and (3) full text was published in English or Chinese.

### Quality assessment

Two investigators independently assessed the methodological quality of each included RCT using the Physiotherapy Evidence Database (PEDro) scale [5]. The 11 items were based on the Delphi list [6]. Each item was scored “+” or “−” with a maximum score of 10 because criterion 1 was not scored. A trial with a score of 6 or more was considered high quality. Conflicts were resolved by discussion with another investigator.

### Data extraction

Both researchers extracted relevant data including study design, sample size, patient age, gender, body mass index, thrombosis prevention, length of follow-up, and all the related complications (wound redness or skin edge necrosis, infection, swelling, and deep vein thrombosis).

### Statistical analysis

Meta-analysis was conducted with Cochrane Collaboration Review Manager 5.0. For continuous data, weighted mean difference (WMD) and 95% confidence interval (CI) were used in this study. The statistical method was inverse variance. For dichotomous outcomes, risk ratio (RR) and 95% CI were calculated as the summary statistics. The statistical heterogeneity was tested with the *χ*^2^ test and *I*^2^ test. *I*^2^ < 25% was considered low statistical heterogeneity, *I*^2^ < 50% moderate statistical heterogeneity, and *I*^2^ < 75% high statistical heterogeneity [7]. If the *P* value of heterogeneity was less than 0.1, heterogeneity would exist. Then, the random-effects model was used for meta-analysis.

## Results

### Search results

The literature search initially yielded 130 relevant trials. There were 104 articles after removing duplicates. We excluded 99 articles on the basis of titles and abstracts, leaving five potentially relevant studies. Nevertheless, one study was a prospective clinical controlled trial, but not a RCT, and the general characteristics of patients were unclear [1]; one study was overlapping with another RCT [8]. Finally, only three RCTs met the predetermined inclusion criteria (Figure 1) [9-11].

**Figure 1:** **Flowchart summarizing the selection process of randomized controlled trials (RCTs).**

Thirty males and 95 females (total, 125 patients) comprised our final study population, with an average age of 65 years (range, 37–84 years). The average follow-up was 14 months (range, 12–28 months). Table 1 shows the characteristics of each included study population. Surgical procedures were conducted by senior orthopedic surgeons.

**Table 1:** **Study characteristics**

**Study**	**Study design**	**Sample size**			**Mean age (years)**	**Gender (M/F)**	**BMI (kg/m** ^**2**^ **)**	**Thrombosis prevention**	**Follow-up(month)**
		**Patients**	**Knees**	**OA**					
Kim YH et al. 1998 [10]	RCT	69	138	84.1%	64 (37–80)	7/62	26	NR	16 (14–28)
Xiong MY et al. 2008 [11]	RCT	16	32	62.5%	65 (45–84)	7/9	26	Aspirin	12
Fan Y et al. 2013 [12]	RCT	40	80	100%	66.5 (49–75)	16/24	NR	LMWH	12

*RCT* randomized controlled trials, *OA* osteoarthritis, *M/F* male/female, *BMI* body mass index, *LMWH* low molecular weight heparin, *NR* not reported.

### Characteristics and quality of included studies

The methodological quality of each included RCT was assessed in accordance with the PEDro scale. The results showed that two RCTs were of high and one trial was of low methodological quality. All the studies used the randomized method. Two studies used concealed allocation. No study used the blinding method. The methodological score of each included trial with general remarks is shown in Table 2.

**Table 2:** **PEDro critical appraisal scores**

**Study**	**PEDro criteria**											**Total**
	**1**	**2**	**3**	**4**	**5**	**6**	**7**	**8**	**9**	**10**	**11**	
Kim et al. [9]	−	+	+	+	−	−	−	+	+	+	+	7
Xiong et al. [10]	−	+	+	+	−	−	−	+	−	+	+	6
Fan et al. [11]	−	+	−	+	−	−	−	+	−	+	+	5

PEDro criteria: 1. Eligibility criteria. 2. Random allocation. 3. Concealed allocation. 4. Baseline comparability. 5. Participant blinding. 6. Therapist blinding. 7. Assessor blinding. 8. >85% follow-up. 9. Intention-to-treat analysis. 10. Between-groups statistical comparison for at least one key outcome. 11. Point estimates and variability measures for at least one key outcome.

### Complications

There were 56 total complications in TKA without drainage and 17 with drainage (Table 3). The forest plot of complication rates indicated statistical difference in TKA between no drainage and drainage (*P* < 0.01, *I*^2^ = 12%) (Figure 2); however, no statistical difference existed when erythema and ecchymosis were excluded (*P* = 0.87, *I*^2^ = 59%) (Figure 3). Besides, there was also no statistical difference in circumference at 10 cm above the patellae on the seventh day after surgery between the two groups (*P* = 0.16, *I*^2^ = 63%) (Figure 4).

**Table 3:** **Results of complications**

**Complications**	**No drainage**	**Drainage**
Erythema/ecchymosis	51	9
Skin edge necrosis	2	4
Deep infection	1	2
Calf muscular venous thrombosis	2	1
Wound redness	0	1
Total	56	17

**Figure 2:** **Forest plot for complication rates with erythema and ecchymosis of bilateral TKA with and without drainage.**

**Figure 3:** **Forest plot for complication rates without erythema and ecchymosis of bilateral TKA with and without drainage.**

**Figure 4:** **Forest plot for circumference at 10 cm above the patellae of bilateral TKA with and without drainage.**

## Discussion

Since the goals of drainage are to prevent hematoma accumulation, to decrease the risk of infection, and finally to obtain a minimum of complications and adverse events, the current study was conducted to objectively evaluate the clinical efficacy and safety of drainage in one-stage bilateral TKA. The most significant finding of the present study was that except for less erythema and ecchymosis around the wound in the drainage group, there were no statistical differences in wound healing, wound infection, swelling, and deep vein thrombosis in one-stage bilateral TKA with and without drainage.

According to a survey of all members of the British Orthopedic Association, 94% of surgeons in the United Kingdom, accounting for 80% of all TKA, used closed suction drainage, and the primary reason was fear of hematoma formation and infection [12]. Thus, infection was analyzed first. The latest retrospective study by Demirkale et al. claimed that non-drainage decreased need for blood transfusion and infection rate in bilateral TKA (510 knees in the non-drainage group versus 454 knees in the drainage group) [13]. However, their results showed that the superficial infection rate of non-drainage and drainage was 1.96% and 4.85%, respectively (*P* = 0.078), and that the deep infection rate was 0.78% and 2.6%, respectively (*P* = 0.111). Besides, there was also no statistical difference in urinary tract infection, pulmonary embolism, and hemarthrosis between the non-drainage and drainage groups (*P* > 0.05) [14]. In addition, several meta-analyses based on unilateral TKA proclaimed no statistical difference in complication rates in TKA with and without drainage [3,4,14], which were consistent with the findings of the current meta-analysis.

There were several strengths of the current study. First, we did a thorough search of the published literature; both English and Chinese full texts were included. Second, all the included studies were RCTs with a low risk of bias.

Some possible limitations to this meta-analysis should be pointed out. First, only three RCTs were included in this current study. There might be a potential publication bias. Second, the total number of patients was too small to have much power as expected. Thus, further multi-center studies with more patients should be performed to have a subjective evaluation of postoperative complications, especially revision rate.

In conclusion, the current evidences confirm that drainage and non-drainage have similar clinical significance and value in one-stage bilateral TKA. However, due to the limitations of the current study, our conclusion should be used with caution. Therefore, future studies with high methodological quality and long-term follow-up periods are needed for updated meta-analyses to better evaluate the clinical efficacy and value of drainage.
